The article "Application of 64-Slice Spiral CT Imaging Technology Based on Smart Medical Augmented Reality in the Diagnosis of Foreign Bodies in the Respiratory Tract in Children" was retracted in 2023. Reasons: signs of a paper mill; suspected computer-generated content; unreliable results or conclusions; lack of ethics approval or compliance.

# Application of 64-Slice Spiral CT Imaging Technology Based on Smart Medical Augmented Reality in the Diagnosis of Foreign Bodies in the Respiratory Tract in Children

**DOI:** 10.1155/2021/9962997

**Published:** 2021-04-28

**Authors:** Jiewei Liu, Ying Wang, Tana Zhao, Chunyu Li, Lei Nie

**Affiliations:** Pediatric Department, The First Affiliated Hospital of Jiamusi University, Jiamusi 154000, Heilongjiang, China

## Abstract

A foreign body in the respiratory tract is one of the common accidental injuries of children in our country, and is usually an important and serious event. Injuries caused by foreign substances in the respiratory tract seriously threaten the health and life of children in Korea and are a great challenge for parents as well. In the process of diagnosis of foreign bodies in the respiratory tract, there is often missed diagnosis or serious complications. Therefore, this article proposes the application of 64-slice spiral CT imaging technology based on smart medical augmented reality in the diagnosis of foreign bodies in the respiratory tract in order to improve the diagnosis of foreign bodies in the respiratory tract, provide help with treatment to improve the prognosis of foreign bodies in the respiratory tract, and reduce the incidence of foreign bodies in the respiratory tract. In this paper, 36 children underwent a 64-slice spiral CT scan of their lungs, and images were transferred to a workstation for multiplanar reconstruction, minimal density projection, three-dimensional volume reconstruction imaging, and CT virtual endoscopic reconstruction, the location, shape, size, and size of the foreign body in contrast with adjacent structural lesions and lesions seen during surgery. Experiments have shown that the left bronchial granulation accounted for 27.3%, the right bronchial granulation 18.75%, the main tracheal granulation 28.6%; there was no significant difference between the left and right bronchial granulation (*P* > 0.05), while the main tracheal granulation and bilateral bronchial granulation there are significant differences between the shape distributions (*P* < 0.05). This shows that CT imaging technology has enabled more patients to avoid surgical operations and ensure that the spiral computer can bring the greatest benefits to children. A 64-slice spiral CT scan can diagnose foreign bodies in the child's respiratory tract. The detection rate is high and the diagnostic failure rate is low. The diagnostic rationale provides a reference for early clinical treatment.

## 1. Introduction

A respiratory foreign body is a common critical illness in the otolaryngology department. It is more common in children under 5 years old and occasionally in adults. It often causes various degrees of breathing difficulties and even death. Therefore, it must be diagnosed as soon as possible and given correct and effective treatment. Therefore, the diagnosis of foreign bodies in the respiratory tract must be clear, and the size, shape, nature, and location of the foreign body must be understood as much as possible. As the continuous advancement of CT imaging technology and its application is gradually pushed forward, the method of obtaining high-quality CT images under conditions of the low signal-to-noise ratio of low-dose scan and projection data has become the focus of interest. Therefore, researchers need to continually improve their CT system hardware and software to meet people's demands for high-quality CT images.

The article "Application of 64-Slice Spiral CT Imaging Technology Based on Smart Medical Augmented Reality in the Diagnosis of Foreign Bodies in the Respiratory Tract in Children" was retracted in 2023. Reasons: signs of a paper mill; suspected computer-generated content; unreliable results or conclusions; lack of ethics approval or compliance.

The diagnosis of respiratory foreign bodies in children using multislice spiral CT imaging technology is much faster than in China, and the development and update of pediatric respiratory foreign bodies diagnosis technology are fast. Methods of diagnosis of pediatric respiratory foreign bodies have been greatly improved and developed. The treatment of multislice spiral CT imaging technology is believed to be an important breakthrough in the near future based on traditional energy integrated detectors [1]. Avramov et al. have carried out CT time subtraction imaging simulation and experimental research on the head model injected with iodine and gadolinium contrast agent. The results show that the time subtraction imaging can make the contrast agent image prominently presented [2]. Kasemsiri et al. believe that the inhalation of foreign bodies in children will cause great pain to children, and the more serious ones may even be life-threatening. He proposed that CT imaging technology can reduce the chance of misdiagnosis or missed diagnosis when diagnosing foreign bodies in the respiratory tract so that more children can be as early as possible and accurately diagnose the foreign body in the respiratory tract [3]. Egorov and Mustafaev and others conducted a questionnaire survey on 1490 mothers of children under the age of 2 to learn their understanding of nut-like respiratory foreign bodies, which proved that parents generally lack the awareness of preventing accidental injury of children's respiratory foreign bodies [4].

The detection and diagnosis of foreign bodies in the pediatric respiratory tract using advanced multislice spiral CT imaging technology began in western countries [5]. The detection and diagnosis of foreign substances in the respiratory tract of children in Korea started clinically late compared to Western countries, and their development is relatively slow. With the continuous development and advancement of modern science and technology and the increasing maturity of medical technology, the use of advanced multistage spiral CT imaging therapy will be an important research work to improve the diagnosis of respiratory foreign bodies in children and to accurately diagnose foreign bodies in the respiratory tract in children. Bogdanova performed image reconstruction on 39 children in the hospital with CT imaging technology [6]. The results of the foreign body exploration and removal under bronchoscope were compared with the results after image reconstruction. The accuracy rate reached 95% [7]. In order to improve the accuracy of the diagnosis of foreign bodies in the airway of children, Mitev MA compares the accuracy of the diagnosis of foreign bodies in the airway of the two groups of children, which proves that the multislice spiral CT imaging technology has a high application value in the diagnosis of foreign bodies in the airway of children and improves the diagnosis [8]. Yildiran and Sunam believe that preventing foreign bodies in a child's respiratory tract is more important than treatment. An in-depth study of the epidemiologic properties of foreign bodies in the airways is very important in preventing such emergencies [9].

The article "Application of 64-Slice Spiral CT Imaging Technology Based on Smart Medical Augmented Reality in the Diagnosis of Foreign Bodies in the Respiratory Tract in Children" was retracted in 2023. Reasons: signs of a paper mill; suspected computer-generated content; unreliable results or conclusions; lack of ethics approval or compliance.

This article aims to deepen the understanding of foreign bodies in the respiratory tract, enhance the understanding of the relationship between the nature of foreign bodies in the respiratory tract and the formation of granulation in the respiratory tract, reduce the misdiagnosis of foreign bodies in the respiratory tract, and improve the prognosis of foreign bodies in the respiratory tract. At the same time, the accuracy of the 64-slice spiral CT imaging technique in diagnosing pediatric respiratory foreign bodies, the type of foreign bodies during diagnosis and confirmation, and the relationship between age and age are studied. To analyze the location of respiratory foreign bodies, we applied 64 slice helix CT imaging technology to diagnose respiratory foreign bodies, allowing the clinic to widely promote this technology so that respiratory foreign bodies can get an accurate diagnosis as soon as possible.

## 2. Application of CT Imaging Technology in the Diagnosis of Foreign Bodies in the Respiratory Tract of Children

### 2.1. X-Ray CT Imaging Principle and Image Reconstruction

#### 2.1.1. X-Ray CT Imaging Principle

(1) The principle of traditional X-ray CT imaging: X-ray CT imaging is an imaging technique that uses certain CT reconstruction algorithms to generate images of the internal structure of the target by measuring the X-rays transmitted through the target [10]. The specific steps of X-ray CT imaging are as follows: First, the continuous X-ray energy spectrum generated in the X-ray tube interacts with the inspected target, and the projection data is generated by analog-to-digital conversion [11, 12]; then, a specific CT reconstruction is used and the algorithm calculates the value of the X-ray attenuation factor absorbed by the object being examined. Finally, the calculated X-ray attenuation coefficient value is transmitted to the computer and converted to the corresponding gray value to obtain a CT image of the object to be examined [13].

The article "Application of 64-Slice Spiral CT Imaging Technology Based on Smart Medical Augmented Reality in the Diagnosis of Foreign Bodies in the Respiratory Tract in Children" was retracted in 2023. Reasons: signs of a paper mill; suspected computer-generated content; unreliable results or conclusions; lack of ethics approval or compliance.

The attenuation characteristics of any substance can be quantitatively expressed by the linear attenuation coefficient *μ*. When a single energy X-ray at specific energy is incident on a target with a uniform density distribution, the attenuation and reduction law obeys Lambert-Beer law, and the number of unattenuated photons *I*_*l*_ can be expressed as follows:

(1) $$\begin{array}{c} I_{l}=I_{0}e^{-\mu l}, \end{array}$$

where *I*_0_ is the total number of incident photons, and *l* is the thickness of the uniformly inspected target.

In medical diagnosis, the actual density distribution of the object being examined is not uniform [14]. When dealing with such a situation, usually the microelement method is used to divide the nonuniform inspection object into *N* small units along the X-ray scanning direction, assuming that the linear attenuation coefficients of each unit are the same. [15, 16]. According to Lambert-Beer's law, the number of photons transmitted through an inspection object can be expressed as follows:

(2) $$\begin{array}{c} I_{l}=I_{0}e^{-\left(\mu_{1}I_{1}+\mu_{2}I_{2}+\cdots +\mu_{N}I_{N}\right)}=I_{0}e^{-\sum \mu_{i}I_{i}}. \end{array}$$

In equation (2), *μ*_1_, *μ*_1_, ⋯, *μ*_*N*_ represents the linear attenuation coefficient of the 1,2, ⋯, *N* small unit object, and *l*_1_, *l*_1_, ⋯, *l*_*N*_ represents the thickness of the 1,2, ⋯, *N* small unit object. When *N* tends to infinity, the integral form of equation (2) can be written as follows:

(3) $$\begin{array}{c} I_{l}=I_{0}e^{-\int \mu \left(l\right)\text{d}l}. \end{array}$$

In equation (3), *μ*(*l*) represents the linear attenuation coefficient of each unit of the nonuniform inspected target along the X-ray path. However, the linear attenuation coefficient of the inspected target is also related to the X-ray energy, which can be expressed by *μ*(*E*, *l*). In medical diagnosis, almost all X-ray sources used are a continuous energy spectrum, covering different energy levels [17, 18]. Then formula (3) becomes as follows:

(4) $$\begin{array}{c} I_{l}\left(E\right)=I_{0}\left(E\right)e^{-\int \mu \left(E,l\right)\text{d}l}. \end{array}$$

In formula (4), *I*_0_(*E*),  *I*_*l*_(*E*), respectively, represent the number of photons before passing through the inspected target and the number of photons that are not attenuated after passing through the inspected target when the energy of the X-ray energy spectrum is the case, ∫*μ*(*E*, *l*)d*l* is the inspected target along the X-ray path *l*; the line integral of the attenuation coefficient [19] is numerically equal to the natural logarithm of the ratio of the number of incident photons to the number of transmitted photons, that is, the projected measurement value *p*, and its expression is as follows:

(5) $$\begin{array}{c} p=\int \mu \left(E,l\right)\text{d}l=\ln\frac{\left(I_{0}\left(E\right)\right)}{I_{l}\left(E\right)}. \end{array}$$

The image reconstruction process is to estimate the linear attenuation coefficient *μ*(*E*, *l*) of the substance through a series of projection measurement values *p* and assign different gray values according to its size to display it in the form of an image [20].

(2) Principles of photon counting X-ray CT imaging: Suppose that the photon intensity of the continuous X-ray energy spectrum generated by the X-ray tube at a certain tube voltage is *I*_0_(*E*), and *T*_1_ is the energy corresponding to the X-ray photon under the continuous energy spectrum. For the set energy threshold *T*_1_, the energy is higher than the energy under the empty scan. The number of photons *I*_*T*_1__ collected by the threshold *E* detector is as follows:

(6) $$\begin{array}{c} I_{T_{1}}=\int_{T_{1}}^{T_{\text{Max}}}I_{0}\left(E\right)\text{d}E. \end{array}$$

In the same way, for the two set energy thresholds *T*_1_, *T*_2_, the number of photons *I*_(*T*_1_, *T*_2_)_ collected by the detector in a specific energy range [*T*_1_, *T*_2_] under empty scanning is as follows:

(7) $$\begin{array}{c} I_{\left(T_{1},T_{2}\right)}=I_{T_{2}}-I_{T_{1}}=\int_{T_{1}}^{T_{2}}I_{0}\left(E\right)\text{d}E. \end{array}$$

When the X-ray photons in the energy section [*T*_1_, *T*_2_] pass through and interact with the inspected target, the number of unattenuated photons *I*_(*T*_1_, *T*_2_)_′ can be expressed by the Lambert-Beer law as follows:

(8) $$\begin{array}{c} I_{\left(T_{1},T_{2}\right)}^{\prime }=I_{\left(T_{1}-T_{2}\right)}e^{-\int \mu \left(E\left(T_{1},T_{2}\right),l\right)\text{d}l}. \end{array}$$

where *μ*(*E*(*T*_1_, *T*_2_), *l*) is the linear attenuation coefficient of the material in the energy section [*T*_1_, *T*_2_] under the X-ray path *l*. When the energy threshold *T*_1_, *T*_2_ is small, the X-ray photons collected by the photon counting detector are approximately monoenergy [21, 22]. Then there are the following:

(9) $$\begin{array}{c} p_{\left(T_{1},T_{2}\right)}=\ln\frac{I_{\left(T_{1},T_{2}\right)}}{I_{\left(T_{1},T_{2}\right)}^{\prime }}=\int \mu \left(E\left(T_{1},T_{2}\right),l\right)\text{d}l. \end{array}$$

Through a series of projection measurements along the X-ray path *l*, a certain reconstruction algorithm is used to estimate the linear attenuation coefficient *μ*(*E*(*T*_1_, *T*_2_), *l*) of the material in the energy section, and the corresponding gray value is assigned according to its size and displayed in the form of an image [23].

The article "Application of 64-Slice Spiral CT Imaging Technology Based on Smart Medical Augmented Reality in the Diagnosis of Foreign Bodies in the Respiratory Tract in Children" was retracted in 2023. Reasons: signs of a paper mill; suspected computer-generated content; unreliable results or conclusions; lack of ethics approval or compliance.

#### 2.1.2. X-Ray CT Image Reconstruction Algorithm

(1) Radon transform and inverse transform: Given a two-dimensional function *f*(*x*_1_, *x*_2_), the corresponding polar coordinate expression is $\hat{f}\left(r,\theta \right)$, where *ϕ* and *u* are the position parameters of the straight line *z*, and the Radon transform and inverse transform expressions are as follows:

(10) $$\begin{array}{c} p=\int_{-\infty }^{+\infty }f\left(x_{1},x_{2}\right)\text{d}z=\int_{-\infty }^{+\infty }\overset{⌢}{f}\left(r,\theta \right)\text{d}z=\int_{-\infty }^{+\infty }\overset{⌢}{f}\left(\sqrt{u^{2}+z^{2}},\varphi +tg^{-1}\frac{z}{u}\right)\text{d}z,\\ \overset{⌢}{f}\left(r,\theta \right)=\frac{1}{2\pi^{2}}\int_{0}^{\pi }\int_{-\infty }^{+\infty }\frac{1}{r\;\cos\left(\theta -\varphi \right)-u}\frac{\partial p}{\partial u}\text{d}u\text{d}\varphi . \end{array}$$

Radon inverse transformation points out that the two-dimensional function *f*(*x*_1_, *x*_2_) can be recovered from a set of countless multiple projection values.

(2) Iterative reconstruction algorithm: Since the iterative image reconstruction algorithm starts from the initial value of the image to be reconstructed, the solution process only needs to solve the forward projection value of the image, and there is no need to find an inverse analysis representation of the projection. If there is no projection data, the image checks the target CT image [24–27]. So the reconstructed image will have a higher image accuracy. The discrete pixel values of the reconstructed image and the projection data collected by the detector can be expressed by the following formula:

(11) $$\begin{array}{c} Ax=p. \end{array}$$

In formula (11), *x* is the image to be reconstructed. If the system transmission matrix *A* is invertible, then there is *x*=*A*^−1^*p*. However, in actual imaging, the system transmission matrix *A* is usually not a square matrix. In this case, the least squares optimization objective function can be used to solve the problem of minimizing the difference between the estimated projection value of the reconstructed image and the actual measured projection value. The specific expression is as follows:

(12) $$\begin{array}{c} \phi \left(x\right)={\left\|Ax-p\right\|}_{2}^{2}. \end{array}$$

The idea of the ART algorithm is to minimize the above objective function so that the iterative formula is as follows:

(13) $$\begin{array}{c} x_{i}^{\left(n+1\right)}=x_{i}^{\left(n\right)}+\lambda_{n}\frac{a_{ij}}{{\left\|A^{j}\right\|}^{2}}\left(p_{j}-A^{j}x_{i}^{\left(n\right)}\right). \end{array}$$

In equation (13), *n* is the number of iterations, ‖*A*^*j*^‖^2^=∑_*i*=1_*A*_*ij*_^2^ is the Euclidean norm of the *j* row of the system transmission matrix *A*, *λ* is the relaxation factor, and *A*^*j*^*x*_*i*_^(*n*)^ is the theoretical projection value.

The article "Application of 64-Slice Spiral CT Imaging Technology Based on Smart Medical Augmented Reality in the Diagnosis of Foreign Bodies in the Respiratory Tract in Children" was retracted in 2023. Reasons: signs of a paper mill; suspected computer-generated content; unreliable results or conclusions; lack of ethics approval or compliance.

After a certain number of single energy X-ray photons interact with the test object, the photons transmitted through the test object are collected by the detector [28]. After interacting with the material for each number of incident photons, there are finally two possible situations. It is received by the detector and not by the detector, so it can be expressed as a binomial distribution in probability theory. When the number of incident photons is sufficiently large, the process can be explained by the Poisson distribution model [29], and the equation is as follows:

(14) $$\begin{array}{c} y_{i}∼\text{poisson}\left\{{\left[Ax\right]}_{i}+n_{i}\right\},\;i=1,2,\cdots ,N, \end{array}$$

where *y*_*i*_ represents the projection data collected by the detector along the *i* path, [*Ax*]_*i*_ is the projection data on the *i* path, and *n*_*i*_ is the system error of the detector unit [30]. The iterative image reconstruction problem can be transformed into how to find the corresponding image *x* to be reconstructed under a known set of measured projection data *y*=(*y*_1_, *y*_2_,…*∞*, *y*_*N*_)^*T*^. The maximum likelihood estimation method can better deal with the above problems. It solves a set of *x* values based on a set of measured projection values *y*, so that the log-likelihood function *L*(*x*) is maximized:

(15) $$\begin{array}{c} L\left(x\right)=\ln\;g\left(\frac{y}{x}\right). \end{array}$$

Because the projection data collected along different paths are independent of each other, the likelihood function *g*(*y*/*x*) can be expressed as follows:

(16) $$\begin{array}{c} g\left(\frac{y}{x}\right)=\prod_{e}^{N}e^{-{\left[Ax\right]}_{i}}\frac{{\left({\left[Ax\right]}_{i}\right)}^{y_{i}}}{y_{i}}=\prod_{e}^{N}e^{-\sum_{j=1}^{M}a_{ij}x_{j}}\frac{{\left(\sum_{j=1}^{M}a_{ij}x_{j}\right)}^{y_{i}}}{y_{i}}. \end{array}$$

Take the logarithm of formula (16) as the objective function to maximize optimization, which is as follows:

(17) $$\begin{array}{c} \hat{x}=\arg\max\left[L\left(x\right)\right]. \end{array}$$

It is difficult to directly find $\hat{x}$ for the above-mentioned nonlinear problem. The specific step is to continuously update the estimated value of each parameter. After each update, the likelihood function is increased, and finally it is approached to the global maximum [31]. To obtain the maximum likelihood parameter estimate, the iterative formula is as follows:

(18) $$\begin{array}{c} x_{j}^{\left(n+1\right)}=\frac{x_{j}^{\left(n\right)}}{\sum_{i=1}^{N}a_{ij}}\sum_{i=1}^{N}\frac{a_{ij}y_{i}}{\sum_{j=1}^{M}a_{ij}x_{j}^{\left(n\right)}}. \end{array}$$

In the formula, *n*=1,2, ⋯ is the number of iterations, and *j*=1,2, ⋯, *M* is the number of discretized pixel units.

The article "Application of 64-Slice Spiral CT Imaging Technology Based on Smart Medical Augmented Reality in the Diagnosis of Foreign Bodies in the Respiratory Tract in Children" was retracted in 2023. Reasons: signs of a paper mill; suspected computer-generated content; unreliable results or conclusions; lack of ethics approval or compliance.

### 2.2. Treatment Methods and Clinical Manifestations of Foreign Bodies in the Respiratory Tract

#### 2.2.1. Treatment of Foreign Bodies in the Respiratory Tract

In most cases, foreign bodies in the respiratory tract must be removed quickly. Those with obvious infection and no obvious obstruction symptoms can also be operated on after anti-inflammatory treatment, especially in children of low age, a short course of the disease, and poor response, especially for timely surgery. For children with severe breathing difficulties on admission, direct laryngoscopy or bronchoscopy should be performed immediately, with or without anesthesia [32, 33]. The appearance of the foreign body must be analyzed before the operation, the same foreign body must be obtained, and the test clamped in vitro, so as to obtain the most suitable instrument and the best removal method, and to predict the possible failure to avoid serious complications [34]. No serious complications should occur.

#### 2.2.2. Clinical Manifestations of Foreign Bodies in the Respiratory Tract

Choose a bronchoscope with a large diameter according to the diameter of the trachea of the child. Foreign body pliers should be selected according to the shape and surface of the foreign body. The foreign body should correspond to different specifications of foreign body clamps according to different sizes. It must be ensured that after the foreign body is clamped by the foreign body clamp, the cross-sectional area cannot be significantly increased. Otherwise, it will be difficult to pass the glottis or easily fall when passing through the glottis, causing serious complications [35, 36].

## 3. Experimental Design of the Application of CT Imaging Technology in the Diagnosis of Foreign Bodies in the Respiratory Tract of Children

### 3.1. Test Subject

In this experiment, 36 children with suspected respiratory foreign bodies admitted to a hospital from July to December 2020 were selected in this experiment. The age of onset and disease course data of these 36 children are shown in Table 1. These 36 children were treated with postprocessing technology and bronchoscopy to remove foreign bodies. During the operation, each trachea, bronchus, and segmental bronchus were carefully examined with the detailed information of the foreign body provided by the preoperative imaging examination—analysis and comparison of intraoperative conditions. The 36 children were divided into 3 groups according to their ages. Among them, 6 were in the 1-year-old group, 24 were in the 1- to 3-year-old group, and 6 were in the older than the 3-year-old group. The types and locations of foreign bodies, the correlation between the position of foreign bodies in the trachea and the granulation, the relationship between the surface and edge of foreign bodies in the respiratory tract and the formation of granulation, and the imaging statistical analysis are analyzed in six aspects [37], so as to understand the application of CT imaging technology in the diagnosis of foreign bodies in the respiratory tract in children.

The article "Application of 64-Slice Spiral CT Imaging Technology Based on Smart Medical Augmented Reality in the Diagnosis of Foreign Bodies in the Respiratory Tract in Children" was retracted in 2023. Reasons: signs of a paper mill; suspected computer-generated content; unreliable results or conclusions; lack of ethics approval or compliance.

### 3.2. CT Scan and Image Reconstruction

All children underwent 64-slice spiral CT (GELightSpeed, General Electric Company) scans of the lungs, and the images were transferred to the workstation for multiplane reconstruction, minimum density projection, volume reconstruction 3D imaging, and CT virtual endoscopic reconstruction to show the location of foreign objects, morphology, size, and adjacent structure lesions, and contrast with the surgical findings.

### 3.3. Image Diagnosis and Evaluation

All images were diagnosed and evaluated by three doctors in the CT imaging room using the double-blind method, and the final diagnosis was obtained by synthesizing the diagnosis results. The number of cases was calculated based on whether a foreign body in the respiratory tract could be clearly diagnosed. The diagnostic criterion for CT films is that the image quality is clear and the bone structure of the larynx is clearly displayed, which does not affect CT diagnosis. CT value measurement: After standardizing and processing the axial image, adjust it to the best level showing a clear extracone fat gap, select the main observation area and healthy side to measure the CT value, and select the secondary data. It is collected for each part and the average is taken for comparison.

### 3.4. Statistical Processing

SPSS23.0 software was used for data processing, and the count data were expressed in percentage (%), *k* is the number of data in this experiment, *σ*^2^ is the variance of all survey results, and *P* < 0.05 indicates that the difference is statistically significant. The formula for calculating reliability is shown in the following equation:

(19) $$\begin{array}{c} a=\frac{k}{k-1}\left(1-\frac{\sum \sigma_{i}^{2}}{\sigma^{2}}\right). \end{array}$$

The article "Application of 64-Slice Spiral CT Imaging Technology Based on Smart Medical Augmented Reality in the Diagnosis of Foreign Bodies in the Respiratory Tract in Children" was retracted in 2023. Reasons: signs of a paper mill; suspected computer-generated content; unreliable results or conclusions; lack of ethics approval or compliance.

## 4. Application of CT Imaging Technology in the Diagnosis of Foreign Bodies in the Respiratory Tract of Children

### 4.1. Evaluation Index System Based on Index Reliability Testing

Here, we perform reliability analysis on all reliability indicators of each object, and the reliability indicators we choose for each object are slightly different. The results are shown in Table 2.

It can be seen from Figure 1 that the data obtained from the imaging statistical analysis of various indicators have a very good effect on this experiment (*α* > 0.8), age and foreign body type, age and respiratory tract foreign body location, foreign body type, and the position, the relationship between the position of the tracheal foreign body and the granulation, and the relationship between the shape of the foreign body and the formation of granulation. The data obtained by the various indicators have an acceptable influence on this experiment (*α* > 0.7), which shows that the CT imaging technology in this paper is used in children. The six indicators selected for the application in the diagnosis of foreign bodies in the respiratory tract are reasonable, which provide a basis for the follow-up experiments.

### 4.2. Based on Inspection Data

#### 4.2.1. Analysis of Age and Foreign Body Types

Here, we first use CT imaging technology to scan the foreign body in the respiratory tract and perform image reconstruction to show the location, shape, size, and adjacent structural lesions of the foreign body, select the appropriate foreign body forceps and remove the foreign body, and perform statistical analysis according to the age group and the type of foreign body. The results are shown in Table 3.

As can be seen in Figure 2, 15.4% of plant-related foreign bodies were suffocated by 1 year old and younger, 12.5% of animals, and metal-plastic minerals. 73.08% of plants 1–3 years old, 50.0% of animals and metal-plastic minerals; 11.5% over 3 years of age suffocate from plant-derived foreign objects; 37.5% of animal and metal plastic minerals. There is a big difference between foreign body choking in young children and older children. The main foreign body in young children is a vegetable foreign body, and the metal and nonmetallic mineral foreign body in older children has increased significantly. The difference is statistically significant (*P* < 0.05).

#### 4.2.2. Analysis of Age and the Location of Foreign Bodies in the Respiratory Tract

Here, we use CT imaging technology to scan the foreign body in the respiratory tract and perform image reconstruction to show the location, shape, size, and adjacent structural lesions of the foreign body, select the appropriate foreign body forceps and remove the foreign body, and perform statistical analysis according to the age group and the location of the foreign body in the respiratory tract. The results are shown in Table 4.

The article "Application of 64-Slice Spiral CT Imaging Technology Based on Smart Medical Augmented Reality in the Diagnosis of Foreign Bodies in the Respiratory Tract in Children" was retracted in 2023. Reasons: signs of a paper mill; suspected computer-generated content; unreliable results or conclusions; lack of ethics approval or compliance.

It can be seen from Figure 3 that after statistics, the number of foreign bodies in the left and right side and main trachea of children over 3 years old is significantly different from the number of foreign bodies in the left and right side and main trachea of children over 3 years old (*P* < 0.05). The proportion of foreign bodies in the trachea and right bronchus was significantly higher than that before 3 years old. There was no significant difference between the left and right side and main tracheal foreign bodies in children before 3 years old (*P* > 0.05).

#### 4.2.3. Analysis of the Type and Location of Foreign Objects

Here, we use CT imaging technology to scan the foreign body in the respiratory tract and perform image reconstruction to show the location, shape, size, and nearby structural lesions of the foreign body, select the appropriate foreign body forceps and remove the foreign body, and perform statistical analysis according to the type and location of the foreign body. The results are as Table 5 shows.

From Figure 4, it can be seen that the distribution of plant foreign matter, animal foreign matter, metal, and nonmetallic mineral foreign matter in the organ is as follows. As a result of statistical analysis, there was no significant difference in the distribution of foreign substances (*P* > 0.05).

#### 4.2.4. The Correlation between the Location of Tracheal Foreign Body and Granulation

Here, we use CT imaging technology to scan the foreign body in the respiratory tract and perform image reconstruction to show the location, shape, size, and nearby structural lesions of the foreign body, select the appropriate foreign body forceps and remove the foreign body, and analyze the correlation between the position of the foreign body in the trachea and the granulation. The results are shown in Table 6.

It can be seen from Figure 5 that the left bronchial granulation accounted for 27.3%, the right bronchial granulation 18.75%, the main tracheal granulation 28.6%, there was no significant difference between the left and right bronchial granulation (*P* > 0.05), while in the main tracheal granulation there is a significant difference in the distribution of bilateral bronchial granulation shape (*P* < 0.05), indicating that the formation of granulation is obviously related to the airflow velocity and the location of the foreign body. The foreign body is not easy to form intratracheal granulation in the position where the airflow is not easy to stay.

The article "Application of 64-Slice Spiral CT Imaging Technology Based on Smart Medical Augmented Reality in the Diagnosis of Foreign Bodies in the Respiratory Tract in Children" was retracted in 2023. Reasons: signs of a paper mill; suspected computer-generated content; unreliable results or conclusions; lack of ethics approval or compliance.

#### 4.2.5. The Relationship between the Surface and Edge of Foreign Bodies in the Respiratory Tract and the Formation of Granulation

Here we use CT imaging technology to scan the foreign body in the respiratory tract and perform image reconstruction to show the location, shape, size, and nearby structural lesions of the foreign body, select the appropriate foreign body forceps and remove the foreign body, and examine the relationship between the surface and edge of the foreign body in the respiratory tract and the formation of granulation. Analysis and the results are shown in Table 7.

It can be seen from Figure 6 that the incidence of granulation with a smooth surface was 16.7%, the incidence of granulation with a rough surface was 23.1%, and the incidence of granulation with a sharp edge was 33.3%, and the difference was statistically significant (*P* < 0.05).

#### 4.2.6. Imaging Statistical Analysis

Figure 7 is a picture of 3 cases of foreign bodies in the respiratory tract scanned by CT imaging technology and image reconstruction. CT imaging technology is used to locate the position and shape of the foreign body and perform bronchoscopy to take the foreign body according to the reconstructed picture. The first in the second case, a 2 cm-long cone-shaped plastic piece was taken out of the right middle bronchus during the operation, which was consistent with the scanning results of CT imaging technology. In the second case, two small pieces of bone fragments were taken out from the left side bronchus during the operation, and the results were compared with CT imaging. The results of the technical scan were consistent; in the third case, the fava bean husk was removed from the left bronchus during the operation, which was consistent with the scan results of the CT imaging technique. This proves that CT imaging technology has enabled more patients to avoid surgical operations, so that foreign bodies in the respiratory tract of children can be accurately diagnosed as soon as possible.

## 5. Conclusions

When the disease is diagnosed, its clinical manifestations are not specific, and a considerable number of parents of children cannot provide a clear history of coughing with foreign bodies. When the foreign body is inhaled, the trachea is blocked, the bronchus causes secondary infection, atelectasis, pneumothorax, etc. Diagnosis of diseases brings difficulties, making imaging examinations particularly important. The type of foreign body choked by children of different ages is different. The distribution of foreign objects in children of different ages is also different. There is no obvious difference in the distribution of foreign bodies in the respiratory tract on both sides, and there is no obvious relationship between the location of the foreign body and the type of the foreign body. At the same time, the formation of granulation in the respiratory tract caused by the foreign body has nothing to do with the release of age, gender, and shape of the foreign body, but is related to the history of the foreign body, the length of the disease course, the location of the foreign body and the roughness and sharp edges of the foreign body's surface. With the maturity of CT imaging technology and the continuous emergence of supporting equipment, the role of spiral computer in the diagnosis and treatment of pediatric respiratory diseases is irreplaceable, and its indications are gradually expanding. Due to its flexibility, flexibility, and intuitiveness, the discovery of airway structure and luminal contents and foreign body removal, lavage treatment, and examination has incomparable advantages in clinical and imaging examinations. Rapid advances in CT imaging technology have allowed more patients to avoid surgery. However, while optimistic about the applicability of spiral computers, you need to fully understand the potential dangers of spiral computers. It is necessary to evaluate the pros and cons of a particular application process to ensure a spiral computer. Computers can have the greatest benefit to children. The 64-slice spiral CT scan for diagnosing respiratory foreign bodies in children can be used as a basis for diagnosis due to its high detection rate and low diagnostic failure rate and provides reference material for early clinical treatment.

The article "Application of 64-Slice Spiral CT Imaging Technology Based on Smart Medical Augmented Reality in the Diagnosis of Foreign Bodies in the Respiratory Tract in Children" was retracted in 2023. Reasons: signs of a paper mill; suspected computer-generated content; unreliable results or conclusions; lack of ethics approval or compliance.

## Figures and Tables

**Figure 1:** Indicator reliability test analysis chart.

**Figure 2:** Analysis chart of age and foreign body type.

**Figure 3:** Analysis of age and the location of foreign bodies in the respiratory tract.

**Figure 4:** Analysis diagram of foreign body type and location.

**Figure 5:** Correlation analysis between the position of foreign body in trachea and granulation.

**Figure 6:** The relationship between foreign body shape and granulation formation.

**Figure 7:** Imaging statistics analysis chart.

**Table 1:** Children's age of onset and course of disease data sheet.

Age	Number of cases (*n*)	Composition ratio (%)	Time	Number of cases (*n*)	Composition ratio (%)
4 months to 1 year	6	16.67	<24 o'clock	7	19.44
1 to 2 years	13	36.11	1 Day to 3 Days	13	36.11
2 to 3 years	11	30.56	3 Days to 1 Week	6	16.67
3 to 4 years	4	11.11	1 Week to 1 Month	8	22.22
Over 4 years	2	5.56	1 Month to 1 Year	2	5.56

**Table 2:** Data sheet of evaluation index system for index reliability testing.

	Very clear	Clear	General	Not clear	Chaotic	Alpha
Age and type of foreign body	3.61	4.48	4.09	0.60	0.13	0.7412
Age and location of foreign objects	3.61	4.24	3.86	0.57	0.36	0.7355
Type and location of foreign body	3.80	3.87	4.24	0.37	0.38	0.7269
Location of foreign bodies and granulation formation	3.51	3.52	4.04	0.34	0.38	0.7145
Foreign body shape and granulation formation	3.74	3.68	4.44	0.44	0.41	0.7342
Imaging statistical analysis	3.62	4.12	4.37	0.80	0.14	0.8641

**Table 3:** Age and foreign body type data sheet.

Group	Plants	Animal	Metal plastic minerals	No foreign matter	Total
Younger than 1 year	4	1	0	1	6
1 to 3 years old	19	3	1	1	24
Older than 3 years	3	1	2	0	6

**Table 4:** Data sheet of age and the location of foreign bodies in the respiratory tract.

Group	Left side	Right side	Main trachea	Bilateral	Glottis	Total
Younger than 1 year	2	3	0	0	0	5
1 to 3 years old	8	10	5	0	0	23
Older than 3 years	1	3	2	0	0	6

**Table 5:** Foreign body type and location data table.

Group	Plants	Animal	Metal plastic minerals	Total
Left bronchus	7	3	1	11
Right bronchus	10	3	3	16
Main trachea	4	2	1	7

**Table 6:** Correlation data table of tracheal foreign body position and granulation.

Group	Have granulation	No granulation	Total
Left bronchus	3	8	11
Right bronchus	3	13	16
Main trachea	2	5	7

**Table 7:** The relationship between the surface and edge of foreign body in the respiratory tract and the formation of granulation.

Group	Have granulation	No granulation	Total
Smooth surface	1	5	6
Rough surface	3	10	13
Sharp edges	1	2	3

## Data Availability

No data were used to support this study.
